The article "An African Ancestry-Specific Allele of CTLA4 Confers Protection against Rheumatoid Arthritis in African Americans" was retracted in 2009. Reasons: results that could not be reproduced; errors in the data; unreliable data; unreliable results or conclusions.

# An African Ancestry-Specific Allele of *CTLA4* Confers Protection against Rheumatoid Arthritis in African Americans

**DOI:** 10.1371/journal.pgen.1000424

**Published:** 2009-03-20

**Authors:** James M. Kelley, Laura B. Hughes, Jeffrey D. Faggard, Maria I. Danila, Monica H. Crawford, Yuanqing Edberg, Miguel A. Padilla, Hemant K. Tiwari, Andrew O. Westfall, Graciela S. Alarcón, Doyt L. Conn, Beth L. Jonas, Leigh F. Callahan, Edwin A. Smith, Richard D. Brasington, David B. Allison, Robert P. Kimberly, Larry W. Moreland, Jeffrey C. Edberg, S. Louis Bridges

**Affiliations:** 1 University of Alabama at Birmingham, Birmingham, Alabama, United States of America; 2 Emory University, Atlanta, Georgia, United States of America; 3 University of North Carolina, Chapel Hill, North Carolina, United States of America; 4 Medical University of South Carolina, Charleston, South Carolina, United States of America; 5 Washington University School of Medicine, St. Louis, Missouri, United States of America; University of Oxford, United Kingdom

## Abstract

Cytotoxic T-lymphocyte associated protein 4 (CTLA4) is a negative regulator of T-cell proliferation. Polymorphisms in *CTLA4* have been inconsistently associated with susceptibility to rheumatoid arthritis (RA) in populations of European ancestry but have not been examined in African Americans. The prevalence of RA in most populations of European and Asian ancestry is ∼1.0%; RA is purportedly less common in black Africans, with little known about its prevalence in African Americans. We sought to determine if *CTLA4* polymorphisms are associated with RA in African Americans. We performed a 2-stage analysis of 12 haplotype tagging single nucleotide polymorphisms (SNPs) across *CTLA4* in a total of 505 African American RA patients and 712 African American controls using Illumina and TaqMan platforms. The minor allele (G) of the rs231778 SNP was 0.054 in RA patients, compared to 0.209 in controls (4.462×10^−26^, Fisher's exact). The presence of the G allele was associated with a substantially reduced odds ratio (OR) of having RA (AG+GG genotypes vs. AA genotype, OR 0.19, 95% CI: 0.13–0.26, *p* = 2.4×10^−28^, Fisher's exact), suggesting a protective effect. This SNP is polymorphic in the African population (minor allele frequency [MAF] 0.09 in the Yoruba population), but is very rare in other groups (MAF = 0.002 in 530 Caucasians genotyped for this study). Markers associated with RA in populations of European ancestry (rs3087243 [+60C/T] and rs231775 [+49A/G]) were not replicated in African Americans. We found no confounding of association for rs231778 after stratifying for the *HLA-DRB1* shared epitope, presence of anti-cyclic citrullinated peptide antibody, or degree of admixture from the European population. An African ancestry-specific genetic variant of *CTLA4* appears to be associated with protection from RA in African Americans. This finding may explain, in part, the relatively low prevalence of RA in black African populations.

## Author Summary

Rheumatoid arthritis (RA) is a systemic autoimmune condition affecting the synovial membranes of diarthrodial joints. The etiology of RA is unclear but is thought to result from an environmental trigger in the context of genetic predisposition. We report that a single nucleotide polymorphism (SNP) (rs231778) in *CTLA4*, which encodes a negative regulator of T cell activation, is associated (*p* = 2.4×10^−28^) with protection from developing RA among African Americans. rs231778 is only polymorphic in populations of African ancestry. Protective alleles such as this one may contribute to the purported lower prevalence of RA in African Americans. Our finding appears to be independent from confounding by linkage with the *HLA-DRB1* shared epitope or by genetic admixture. Furthermore, we did not replicate associations of *CTLA4* SNPs with RA or other autoimmune diseases previously reported in Asians and Caucasians, such as rs3087243 (+60C/T) and rs231775 (+49A/G). The associations of different SNPs with RA susceptibility specific to different populations highlight the importance of CTLA4 in the pathogenesis of RA and demonstrate the ethnic-specific genetic background that contributes to its susceptibility.

## Introduction

Cytotoxic T-lymphocyte associated protein 4 (*CTLA4*, CD152) is a negative regulator of T-cell activation. As the T-cell activation signal propagates due to costimulatory B7 molecule (CD80, CD86) binding of CD28, cell surface expression of CTLA4 increases to compete with CD28 [1]. CTLA4 also prevents further clonal expansion of effector T-cells, including regulatory T cells (T_reg_) [2],[3], and can inhibit osteoclast formation [4].

Genetic variation in *CTLA4* (Chromosome 2q33) could contribute to unchecked T cell or osteoclast activation with resultant onset of autoimmune disease such as rheumatoid arthritis (RA). *CTLA4* was modestly associated with RA in a recent genome wide association study (GWAS) of RA in Caucasians [5]. *CTLA4* single nucleotide polymorphisms (SNP), such as rs231775 (+49A/G), have been associated with multiple autoimmune conditions including RA, Addison's disease, autoimmune pancreatitis [6], autoimmune thyroid disease, celiac disease, chronic inflammatory arthritis [7]. multiple sclerosis [8], type I diabetes mellitus, Sjögren's syndrome [9], and systemic lupus erythematosus (SLE) [10]. An association with another SNP, rs3087243 (+60C/T), and RA was found in a Chinese Han population [11]; however, these results were not replicated in Irish [7], United States Caucasian [12], or, when corrected for multiple testing, British Caucasian [13] populations. Analysis of a much larger group of Caucasians from North America and Sweden associated this marker with RA [particularly with the anti-cyclic citrullinated peptide (anti-CCP) antibody positive RA subset] [14]. Given the association of *CTLA4* with multiple diseases in various populations, we sought to characterize the genetic contribution of *CTLA4* to RA in African Americans – a population not yet explored.

RA is purported to be less prevalent in African Americans than in Caucasians based on clinical observation and data in black continental Africans [15]–[19]. African-specific protective alleles might explain the lower disease prevalence among persons of African ancestry and should be evaluated in genetic studies with this population.

In this study, we genotyped *CTLA4* haplotype tagging SNPs (htSNPs) in two groups totaling 505 African American patients with RA and 712 African American healthy controls. We found and replicated a novel protective association at an ethnic-specific intronic SNP, rs231778, in both independent groups. While this SNP is polymorphic only in the HapMap Yoruba population, we confirmed a lack of variation by genotyping 530 Caucasians. Importantly, we did not detect significant confounding for association of rs231778 when our patients were stratified by level of European admixture or by RA subclassification such as presence of the *HLA-DRB1* shared epitope (SE) or anti-cyclic citrullinated peptide (anti-CCP) antibodies [20]. We also did not find association with two SNPs (rs3087243 and rs231775) previously reported to have disease associations with RA in European ancestry populations or with other autoimmune diseases.

Our data reveal a protective African ancestry-specific allele that may contribute to the purportedly lower prevalence of RA in persons of African ancestry and provide suggestions for future research into the relationship between T cell regulation and RA pathogenesis.

## Methods

The Consortium for the Longitudinal Evaluation of African Americans with Early Rheumatoid Arthritis (CLEAR) Registry enrolled self-identified African Americans with RA who met the American College of Rheumatology (ACR) 1987 diagnostic criteria [21]. Participants for CLEAR were recruited from the University of Alabama at Birmingham (UAB) [coordinating center]; Emory University/Grady Hospital (Atlanta, GA); University of North Carolina at Chapel Hill; Medical University of South Carolina (Charleston, SC); and Washington University (St. Louis, MO). Recruitment occurred in two phases: enrollment of patients with early RA (<2 year disease duration) followed longitudinally until 5 years disease duration, from 2000 to 2007 (CLEAR I); and enrollment of patients with RA of any duration from the same sites as part of a cross-sectional analysis from 2007 to present (CLEAR II). Comprehensive demographic, clinical, and radiographic data are being collected on all CLEAR participants, and serum and DNA samples are being stored [22]. These data allow for stratification of RA patients [20] by presence of the *HLA-DRB1* SE and anti-CCP antibody positivity. We have also measured estimated global admixture using a panel of ancestry informative markers (AIMs), as previously reported [23]. A group of healthy African American controls, for the longitudinal arm of this study, with similar sex, age, and geographic location has been recruited, as previously described [23]. All participants were recruited with informed consent under the approval of each respective Institutional Review Board. Genomic DNA was isolated using standard methods and stored at −70°C.

This study included 282 African American RA patients and 149 African American controls from the CLEAR longitudinal study (CLEAR I) and 223 African American RA patients from the CLEAR cross-sectional study (CLEAR II). We also obtained DNA samples from an additional 563 healthy African Americans from Alabama recruited for a case-control study of SLE [24] to use as controls for the CLEAR II RA patients. Demographics for CLEAR I and CLEAR II RA patients are presented in Table 1. Controls were younger than the RA patients (mean age: CLEAR I = 45±14 years, CLEAR II = 35±11 years). Similar to the patient groups, both of the control sets were predominantly female (percent female: CLEAR I = 82%, CLEAR II = 74%). In total, we analyzed 505 African American RA patients and 712 African American controls. We used RA patients and controls from CLEAR I as an initial test set and RA patients from the CLEAR II and additional Alabama controls as a replication group.

**Table 1:** Demographics of populations used in this study.

	CLEAR I (Longitudinal) [n = 282]	CLEAR II (Cross-Sectional)[n = 223]	P value
Age at onset, average (±SD)	55.6 (±13.3)	57.5 (±11.2)	NS
% Female	82.2	86.3	NS
Disease Duration (yrs), mean (±SD)	1.6 (±0.6)	5.9 (±1.6)	<0.0001*
Rheumatoid Factor Positive	72.8	80.3	NS
Anti-CCP Antibody Positive	62.0	60.8	NS
% HLA-DRB1 Shared Epitope Positive	42.7	39.2	NS

Anti-CCP – anti-cyclic citrullinated peptide; SD – standard deviation; NS – not significant. * Inclusion criteria were <2 years disease duration for CLEAR I and any disease duration for CLEAR II.

All SNPs within the *CTLA4* region (±2 kb) that have a minor allele frequency (MAF) ≥0.05 in the Yoruba HapMap population (Phase II/Release 21) were genotyped: rs231775, rs231776, rs231777, rs231778, rs231779, and rs3087243. Data from the resequencing of *CTLA4* in both African and European populations contracted to SeattleSNP (Dr. Debbie Nickerson, University of Washington) were kindly provided from the Population Genetics Study coordinated at UAB (Drs. Richard Kaslow and Robert Kimberly). *CTLA4* SNPs detected by SeattleSNP that capture information on polymorphisms not present in HapMap for Africans with a MAF ≥0.05 were additionally genotyped: rs11571319, rs231772, rs231780, rs34031880, rs733618, and *5251. *5251 is not yet listed in dbSNP: its physical location is 54945227 in NCBI contig file NT_005403, and its surrounding sequence is ATGGTAGCCTTGCTTATTGT [G/T] GGTGGCAACCTTAATAGCAT.

Genotyping was performed by the Illumina FastTrack GoldenGate BeadXpress genotyping service (San Diego, CA) for CLEAR I for SNPs from the International HapMap Consortium. All other genotyping was performed using Applied Biosystems TaqMan Allelic Discrimination Assays (Foster City, CA) on an ABI 7900HT Genetic Analyzer. Overall, between both platforms for all SNPs, our genotyping success rate was 99.4%. We successfully genotyped rs231778 among 74 samples using both platforms with 100% reproducibility. To confirm the monomorphic nature of rs231778, we genotyped this SNP in 530 Caucasian samples from the UAB Treatment of Early Aggressive Rheumatoid Arthritis (TEAR) study.

Fisher's exact tests were performed on SAS 9.0 (Cary, NC) and exact logistic regression tests performed on LogXact 8.0 (Cambridge, MA). We controlled for potential confounding by *HLA-DRB1* status, anti-CCP antibody positivity, and genetic admixture following the approach of Redden et al. [25]. Linkage Disequilibrium and haplotype analyses were performed with HaploView v3.31 [26]. All SNPs were in Hardy-Weinberg Equilibrium (tested with Chi squared tests), except rs231776 (HWE *p* = 0.0085), which was excluded from further analysis.

## Results

### Resequencing and Description of Genetic Variation in CTLA4

Data available from the International Haplotype Mapping Consortium (HapMap), as accessed in February 2008, appear incomplete with regard to coverage of *CTLA4*. Only SNPs present from the 5′ region through intron 1 (rs231775, rs231776, rs231777, rs231778, rs231779) are represented with detailed genotyping data. HapMap does not provide data for SNPs among the remaining exons and introns of *CTLA4* but does present information for polymorphisms in the 3′ end of the gene, such as rs3807243. To select htSNPs that cover the remaining interior portions of this gene, we accessed resequencing data available from SeattleSNP that provided detailed genotypes on YRI and CEU populations. SeattleSNP routinely resequences only 500 basepairs into each end of a given intron. A portion of intron 1 (the longest intron) is the only region of *CTLA4* not completely resequenced by SeattleSNP; however, intron 1 was completely covered by HapMap, allowing the combination of these two resources to provide the most detailed haplotype tagging strategy for this gene. See Figure 1.

**Figure 1:** Only SNPs genotyped in this study are listed by name. SNPs in linkage disequilibrium with SNPs genotyped in this study are shown in brown. SNPs in gray were not genotyped or haplotype tagged due to low minor allele frequency (MAF). SNP - Single Nucleotide Polymorphism. 5251* is not yet registered in dbSNP as described in the methods.

Due to the limited public information on *CTLA4* in African Americans, we used HaploView to calculate linkage disequilibrium (LD) across all genotyped SNPs. A plot representing the LD (r^2^ values) of SNPs is included as Figure 2.

**Figure 2:** This plot, generated from HaploView v3.31 (Broad Institute), shows the r^2^ values between SNPs genotyped in *CTLA4*. Darker boxes represent stronger r^2^ values. 5251* is not yet registered in dbSNP as described in the methods.

### Association of rs231778 with Rheumatoid Arthritis in African Americans

We detected a protective effect for RA in African Americans with the G allele of rs231778 in both CLEAR study groups (longitudinal and cross-sectional) independently and together (CLEAR I and CLEAR II combined Fisher's exact *p* = 4.46×10^−26^). See Table 2. Because homozygotes for the G allele were rare, we compared the frequency of persons with genotypes GG and AG to those with genotype AA. From the odds ratios of the two groups combined, it can be seen that the presence of the G allele confers a protective effect (OR = 0.19, 95% CI: 0.13–0.26, *p* = 2.4×10^−28^, Fisher's exact). See Table 3. rs231778 is not in LD with any other SNP, which suggests any genetic effect it confers is likely independent. See Figure 2.

**Table 2:** Association with rheumatoid arthritis at rs231778 in African Americans.

Genotype		AA	AG	GG	All	Fisher's Exact P value
Longitudinal	RA	249 (0.90)	25 (0.09)	2 (0.01)	276	1.572×10^−8^
	Controls	99 (0.67)	44 (0.30)	4 (0.03)	147	
Cross-sectional	RA	186 (0.89)	21 (0.10)	1 (0.01)	208	5.093×10^−14^
	Controls	324 (0.59)	202 (0.37)	24 (0.04)	550	
Combined	RA	435 (0.90)	46 (0.10)	3 (0.01)	484	4.462×10^−26^
	Controls	433 (0.62)	236 (0.34)	28 (0.04)	697	

Values indicate number of samples with allele frequency in parentheses. Analysis compares number of patients and controls for each genotype (AA vs AG vs GG) in a 3×2 Fisher's exact test.

**Table 3:** Odds ratios for the protective effect of the rs231778 G allele in African Americans with RA.

	OR	95% CI	Fisher's Exact P value
Longitudinal	0.23	0.13–0.39	2.127×10^−8^
Cross-sectional	0.17	0.10–0.28	3.354×10^−17^
Combined	0.19	0.13–0.26	2.437×10^−28^

Analysis compares number of patients and controls for genotype AA vs those with either AG or GG in a 2×2 Fisher's exact test. OR – odds ratio; CI – confidence interval.

The G allele of rs231778 is relatively specific for African populations as only the A allele is detected among Asians and Caucasians genotyped in the International HapMap Project and in Caucasians genotyped by SeattleSNP. Since variation at rs231778 was not found in the HapMap (n = 24) or Perlegen (n = 60) based European samples, we genotyped an additional 530 self-identified Caucasians to assess ethnic specific variation at this site. Among these 530 subjects, only 3 were heterozygous at rs231778, and none were homozygous for the G allele, which yields a MAF of 0.0028. In the 697 healthy African American individuals we genotyped, the MAF is 0.209 illustrating the ethnic specificity of this marker.

Since the presence of the SE has been associated with susceptibility to RA in our population [23] and known to confound association with RA at other immunologically relevant loci such as *PTPN22* [27], we evaluated our findings in *CTLA4* for possible confounding by the HLA-DRB1 SE, the strongest known genetic risk factor for RA. We found that the MAF of rs231778 was not different within cases or controls when stratified for number of SE alleles present. Because only 4 control samples have two SE alleles, we cannot rule out any possible influence of the SE on the genetic contribution of *CTLA4* in RA susceptibility, but it appears to be unlikely. See Table 4.

**Table 4:** Minor allele frequency (MAF) of rs231778 segregated by HLA-DRB1 shared epitope status.

	0 SE Alleles	1 SE Alleles	2 SE Alleles	Total
Patients	0.05 (N = 12/274)	0.06 (N = 9/160)	0.06 (N = 2/34)	0.05
Controls	0.21 (N = 27/130)	0.21 (N = 8/38)	0.25 (N = 1/4)	0.21

This table combines samples from both CLEAR I and CLEAR II and only incorporates data where HLA-DRB1 shared epitope (SE) status has been determined. The ‘N’ listed below each MAF represents the number of ‘G’ alleles over the total number of alleles for each number of SE alleles present. SE – *HLA-DRB1* shared epitope.

Since our study focuses on African Americans, a group with known recent population admixture [28], we assessed percentage of European admixture as a confounding factor in the association of RA with rs231778. Data from a genome-wide admixture panel performed at the Broad Institute from our previously reported work [23] allowed calculations of global admixture estimates (percent European ancestry) for 282 cases and 94 controls (total N = 366). Of these 366 with admixture data, there was successful genotyping for the *CTLA4*-containing region of Chromosome 2 in 266 cases and 81 control samples (total N = 347). We show the mean percentage of European ancestry segregated by genotype for cases and controls in Table 5. The degree of admixture was not associated with rs231778 genotype (Fisher's exact *p* = 0.2367). We confirmed that admixture difference between cases and controls was not significant using the robust Welch test, which produced a value of 2.308 (degrees of freedom = 215.578, *p* = 0.130).

**Table 5:** Mean percentage of European ancestry segregated by genotype of rs231778.

Genotype	AA	AG or GG	AA, AG, or GG
Case	0.172 (0.0997) N = 240 [246]	0.114 (0.062) N = 26 [27]	0.166 (0.098) N = 266 [273]
Control	0.146 (0.052) N = 67 [75]	0.169 (0.078) N = 14 [18]	0.150 (0.057) N = 81 [93]
Total	0.166 (0.092) N = 307 [321]	0.133 (0.072) N = 40 [45]	0.162 (0.090) N = 347 [366]

This table provides data for the 347 samples with complete admixture and rs231778 genotyping data. Standard error is provided in parenthesis. Brackets indicate frequency counts used in determining association of the rs231778 G allele with rheumatoid arthritis among 366 samples, as described in the text.

We did not find a significant association with RA of the G allele among the 347 samples with complete admixture data and *CTLA4* genotypes (asymptotic *p* = 0.0674); we suspect that this is due to the reduced statistical power of analysis of a smaller number of subjects and controls. When we based calculations upon the 366 samples used in our previous admixture-based manuscript [23], this small increase in sample size regained statistical significance of association with RA (asymptotic *p* = 0.0183). To illustrate further the lack of significance among the 347 samples is due to lack of power, frequency counts of genotypes among the 366 samples are incorporated in Table 5 to demonstrate a similar pattern of genotype distributions with and without these additional samples.

### Lack of Genetic Associations with RA at Other *CTLA4* Loci

Nonsynonymous SNPs previously associated in other populations and autoimmune phenotypes (rs3087243 and rs231775) were not associated with RA in our study. See Table 6. We also found no association when we analyzed data based upon deduced haplotypes or at any individual SNP when stratified by RA subclassification (SE status, anti-CCP antibody status, or percent European ancestry) as has been observed with RA associations at other sites in the genome [23] and with *CTLA4* SNPs in Caucasian populations [14]. See Table 6.

**Table 6:** Minor allele frequencies of CTLA4 SNPs for African American RA patients and controls.

SNP	Minor Allele	Position	CCP+ Patients	CCP− Patients	SE+ Patients	SE− Patients	All Patients	Controls	Public Database: African	Public Database: European	Fisher's Exact P values
rs733168	C	−1722	0.134	0.128	0.158	0.113	0.123	0.142	0.15	0.07	0.0113
rs231772	A	−1113	0.030	0.031	0.034	0.033	0.028	0.053	0.09	0.00	0.0462
rs231775	G	48	0.424	0.392	0.442	0.381	0.413	0.372	0.42	0.39	0.2827
rs231776	A	184	0.023	0.031	0.034	0.026	0.027	0.038	0.10	0.00	0.0418
rs231777	T	922	0.240	0.232	0.252	0.238	0.244	0.220	0.13	0.27	0.7651
**rs231778**	**G**	**1155**	**0.053**	**0.046**	**0.063**	**0.046**	**0.054**	**0.209**	**0.09**	**0.00**	**4.462×10^−26^**
rs231779	T	1821	0.464	0.448	0.490	0.424	0.460	0.452	0.42	0.38	0.3718
5251*	A	2107	0.060	0.041	0.034	0.066	0.045	0.040	0.08	0.00	0.8275
rs231780	G	4031	0.082	0.119	0.102	0.096	0.097	0.124	0.17	0.00	0.0667
rs34031880	C	6222	0.036	0.067	0.054	0.043	0.045	0.063	0.04	0.00	0.2222
rs3087243	A	6253	0.161	0.186	0.170	0.169	0.167	0.195	0.17	0.41	0.6343
rs11571319	A	6272	0.217	0.180	0.199	0.215	0.197	0.141	0.12	0.20	0.0731

This table represents combined data from CLEAR I and CLEAR II. rs3087243 (+60C/T) has been associated with RA in Caucasians, and rs231775 (+49A/G) has been associated with other autoimmune conditions. Position is the physical location of each polymorphism relative to the start codon (position = 0) in dbSNP build 129. CCP refers to anti-cyclic citrullinated antibody status. SE refers to presence of HLA-DRB1 shared epitope. Public databases include allele frequencies from HapMap or SeattleSNP. rs231776 was not in Hardy-Weinberg Equilibrium. *5251 is not currently listed in dbSNP as described in the methods.

We found no significant association with the G allele of rs3087243, even when stratified for presence of anti-CCP antibody, as previously reported in Europeans with RA [14]; the distribution of genotypes and allele frequencies of this SNP were similar in anti-CCP antibody-positive and anti-CCP antibody-negative RA patients. Similarly, we found no significant differences in allele frequency between anti-CCP positive RA patients and anti-CCP negative RA patients at the SNP associated with RA in our study (rs231778).

In the initial analysis of the CLEAR longitudinal arm, we found a protective effect (lower allele frequency in patients than controls) of the minor allele (G) of rs231780 allele (Fisher's Exact *p* = 0.0123). However, upon replication in the CLEAR cross-sectional arm, this difference in MAF between cases and controls was not significant in the cross-sectional arm or in both arms combined [Fisher's exact *p* = 0.0667; MAF 0.097 in patients, 0.124 in controls]. See Table 6. Of note, the rs231780 SNP appears to be African-ancestry specific as well, with a MAF of 0.17 in Africans and ∼0.00 in Europeans among HapMap subjects. It is possible that our lack of association at this marker is due to a true negative state or due to lack of power for detecting a positive association, as our the p value is bordering on significance (*p* = 0.07). Although rs231780 is also an ethnic-specific SNP, there is not significant LD between it and the strongly associated SNP rs231778 (r^2^ = 0.107, D′ = 0.445). The lack of association of the African-specific SNP, rs231780, with RA might be sufficient to rule out genetic admixture as the cause of the association at rs231778.

We also found an association with rs231776 (Fisher's exact *p* = 0.0418) when both study groups were combined; however, this SNP was not in Hardy-Weinberg equilibrium (HWE *p* = 0.0085), complicating interpretation of these results.

## Discussion

We detected a significant novel genetic association with RA in African Americans at the *CTLA4* SNP rs231778. In this case-control study, African Americans with at least one minor (G) allele were 0.19 times as likely to have RA as those without a minor allele (95% CI 0.13 0.26, Fisher's Exact *p* = 2.437×10^−28^). This P value does not appear to be subject to the inaccuracy introduced by cancellation error by complementation [29]. Our study is limited in sample size due to its exclusive focus on a minority population, which may introduce influence by bias in sample collection, genotyping errors, and lack of power. However, due to our efforts in matching patients and controls and validating our genotyping results (100% reproducibility in 74 samples on different genotyping platforms), we believe such biases have been minimized. We believe that our study is sufficiently powered to detect associations as we found a statistically significant result in two separate arms of the study.

The associated SNP, rs231778, is located in intron 1 and is not in LD with any genotyped SNP in *CTLA4* such as the disease-associated rs3087243 and rs231775 markers. See Figures 1 and 2. It is possible, however, that LD could span farther than assessed in this study allowing the possibility that rs231778 is a surrogate marker for another associated polymorphism well outside of the gene boundaries of *CTLA4*. LD has been shown to span several megabases in African Americans, which supports this possibility [30]. Additional genotyping of 5–10 AIMs in this chromosomal region in a large number of African Americans may allow a better understanding of the long-range haplotype structure. Our study did include five African-specific SNPs (rs231772, rs231776, rs231780, rs34031880, 5251*) and one AIM, defined as a difference in MAF >0.20 between populations, (rs3087243) that did not associate with RA. The association of the African-specific allele of rs231778 and RA and the lack of association at these ethnic-specific markers supports the idea that the association of rs231778 is independent from bias by genetic admixture.

Interestingly, rs231778 is monomorphic in both Asian and Caucasian populations, according to genotype data from HapMap and SeattleSNP, and virtually absent in our genotyping of 530 Caucasians. Given the ethnic-specific status of this SNP, it is possible that our finding helps to explain the purported, but as yet unproven, observation of a lower prevalence of RA in African Americans compared to Caucasians. We would anticipate the association of such African-specific protective alleles with resistance to RA. Racial or ethnic differences have now been suggested in the association of RA with several genes, including *PTPN22* [31], *PADI4* [32], *SLC22A4* and *RUNX1* [33], and in *CTLA4*, particularly between Asian and Caucasian populations [10],[34]. These data highlight the need for additional research into the genetic background of RA in various populations such as African Americans to uncover additional ethnic-specific associations.

Our study included 697 healthy African American controls that possessed a MAF of 0.209 at rs231778. This finding is surprising since public resources such as the International HapMap Consortium has a MAF of 0.09 in their panel of 60 Yorubans and 0.00 in 60 Caucasians. African Americans are considered to be an admixed population with an African background and contribution of approximately 20% European genetic ancestry. In fact, we calculated that European ancestry contributes 15±5% of the genetic composition of African Americans in the CLEAR study. Therefore, we would expect a MAF for rs231778 to be between 0.00 and 0.09. Given that our participants were collected at multiple centers across the Southeastern United States (with each center having similar MAFs), that we genotyped 74 samples with 100% reproducibility on dual platforms (TaqMan and Illumina), and that our study included a larger number of samples (n = 697) than public resources (n = 60), we believe our results are accurate. Such a difference from the expected MAF may be due to reduced power in HapMap compared to this work or due to population stratification (i.e. the MAF of 0.09 for Yorubans in Nigeria could be markedly lower than elsewhere on the continent from where ancestors of our participants may have lived). More work into the genetic population structure across Africa and in admixed populations such as African Americans is needed to appreciate such differences.

Population-based differences in susceptibility to RA are observed through previous reports that show an association between RA and rs3087243 (+60C/T), a polymorphism known to affect the expression levels of soluble CTLA4 protein [35], in Swedish and North-American populations [14] or a lack of association at this locus in studies based in Massachusetts or Northern Ireland [7],[13]. We failed to find an association of rs3087243 in RA among African Americans. Even when stratifying for a clinical subclassification more strongly associated with *CTLA4* [14] (anti-CCP positivity), we could not reproduce these results in African Americans. This non-replication finding may be due to genuine population-specific differences in allele frequency or different patterns of LD among African and European ancestry individuals, but our relatively small sample size precludes definitive conclusions. For example, to detect a small genetic effect [OR = 1.08 (95% CI: 1.01–1.17)] in a meta-analysis of genotypes, Plenge et al. analyzed ∼4,000 Caucasian RA samples [14], a much higher number of subjects than is available for our analysis. We also failed to find an association with the nonsynonymous SNP, rs231775 (+49A/G), which has been implicated in multiple autoimmune diseases, again possibly due to small sample size.

CTLA4 is an important molecule in preventing an inappropriate immune response and in dampening osteoclast formation [4], both of which may have implications for the pathogenesis of RA. CTLA4 stimulation functions in regulatory T cell development including proliferation and frequency [2],[3],[36], providing another possible mechanism for this protein to influence RA pathogenesis. While we do not address possible functional consequences of this polymorphism, future work may reveal a relationship between rs231778 and T cell/osteoclast development or linkage disequilibrium with a SNP outside of the CTLA4 gene boundaries that influences expression or function.

In conclusion, our results suggest a need for greater understanding of CTLA4 function and of the ethnic-specific genetic contributions to RA including relationship to disease pathogenesis.
